The article "PSO Algorithm-Based Design of Intelligent Education Personalization System" was retracted in 2023. Reasons: signs of a paper mill; suspected computer-generated content; unreliable results or conclusions; concerns about the data.

# PSO Algorithm-Based Design of Intelligent Education Personalization System

**DOI:** 10.1155/2022/9617048

**Published:** 2022-07-09

**Authors:** Pengjiao Li, Jun Yang

**Affiliations:** College of Educational Science, Bohai University, Jinzhou 121000, Liaoning, China

## Abstract

The application of artificial intelligence in the field of education is becoming more and more extensive and in-depth. The intelligent education system can not only solve the limitations of location, time, and resources in the traditional learning field but it can also provide learners with a convenient, real-time, and interactive learning environment and has become one of the important applications in the Internet field. Particle swarm optimization (PSO) is a swarm intelligence-enabled stochastic optimization scheme. It is derived from a model of bird population foraging behavior. Because of its benefits of ease of implementation, high accuracy, and quick convergence, this algorithm has gained the attention of academics, and it has demonstrated its supremacy in addressing real issues. This paper aims to study the optimization of PSO in the field of computational intelligence, improve the matching degree of learning resource recommendation and learning path optimization, and improve the learning efficiency of online learners. This paper suggests intelligent education as the center, takes the PSO algorithm as the main research object, and expounds the related concepts of intelligent education and PSO algorithm. It uses swarm intelligence algorithms for intelligent education personalized services. He focuses on PSO algorithm and its work in intelligent education recommendation and learning path planning. Experiments show that the average value of the difference between the two obtained by the NBPSO algorithm is 1.13*E* + 02 and the variance 1.88*E* + 02 is the smallest. Therefore, PSO aids in improving the quality and consistency of online course resource development. In conclusion, the research results of this paper further demonstrate the advantages of PSO algorithm in solving the problem of personalized service in intelligent education. It can promote the in-depth application of swarm intelligence optimization algorithms in intelligent online learning systems. This effectively enhances the intelligent service level of the online learning system and increases the efficiency of online learning.

## 1. Introduction

Currently, with the constant advancement of China's education reform, the educational model of education is quietly changing. An intelligent education system is particularly important for colleges and universities. Emerging technologies represented by cloud computing, mobile Internet, machine learning, big data, and computational intelligence are booming. It has not only considered as a vital driving force for global industrial upgrading and transformation but also created application scenarios across time and space. Moreover, it is profoundly changing the way of human learning and promoting the deep integration and development of artificial intelligence and educational applications [1]. The PSO algorithm originated from the study of simple life groups [2]. Now the PSO algorithm has been well expanded and applied in many aspects, intelligent education is one of them. The advent of PSO has made many scientists shine, this algorithm is a new group optimization algorithm. Its main feature is that it does not require too many parameters, nor does it require too much knowledge, nor does it require very complicated principles. Its convergence speed is also very fast, which makes the problems caused by traditional optimization algorithms easily solved.

The research of intelligent education has strong application and urgent demand of the times, which is of unlimited importance to the development of online intelligent education. In the context of the vigorous development of “Internet +” educational applications, this paper attempts to start with the research on the personalized system of intelligent education. It uses computational intelligence optimization algorithms to solve and analyzes the characteristics of intelligent education. It improves the learning efficiency of intelligent education through the optimization research of computational intelligent particle swarm algorithm. It explores the online learning resource serialization service mechanism and builds a relatively complete theoretical system of intelligent education serialization service. For educational departments or sections, universities and colleges, management system, particularly intelligence and information based, is also a key topic. Intelligent education has the potential to not only increase the efficiency of school teaching departments, but also to encourage the development of intelligent, information-based, and digital campuses.

The innovation of this paper is that: (1) it applies PSO to the learning algorithm of radial basis NN. It is mainly a learning procedure or technique or algorithm for function approximation, and the P-RBF algorithm is proposed. (2) In this paper, the radial basis NN in the NN is studied, and the particle swarm algorithm is applied to the research of designing the individualization of intelligent education. This method has good practicability and accuracy in online learning path optimization.

## 2. Related Work

With the wide application of PSO in various fields, it has become a research hotspot of the majority of scientists. In India, the literacy rate of deaf students is very low, and an effective academic prediction model is needed to identify deaf students. The research of Durga and Jeyaprakash found that the regression model established by NN has long convergence time and high error rate. To address the NN's issue, the PSO approach is utilised to change the weights of the NN. The choice of starting parameters is, however, one of the key drawbacks of the PSO method. As a result, Durga and Jeyaprakash introduce a novel PSO technique that use the regression formula to establish the NN's initial weights. The findings reveal that the NN built with this approach performs better than the NN built with the basic PSO algorithm. This study's mean squared error is 0.0998, which is lower than several previous models [3]. When the allowable space of state for UAVs is severely limited, a method for picking space of state is more efficient than control space's sampling. While this is self-evident, the practical problem is figuring out how to do so while staying within the dynamic feasible constraints of the vehicle. Daryina and Prokopiev provide a deep convolutional NN (CNN) for real-time picture interpretation based on a predictive integrated path model (MPPI) controller. He also suggested a PSO UAV control technique for determining the cost function parameter vector that is optimum. The technique is based on a cost function that defines where the vehicle should proceed on the path surface [4]. Renewable energy (RE) systems are important in the production of power all over the world. The autonomous hybrid microgrid (A-HMG) technology is used to integrate the RE system from the distributed side. The A-HMG idea includes a number of technological solutions that must be managed effectively. Mouachi et al. propose using the multimodal delay PSO, a novel nature-inspired meta-heuristic optimization method, as a solution (MDPSO). He used the method to A-HMG and discovered the lowest levelized energy cost, the lowest chance of power loss, and the highest renewable coefficient [5]. In his study, Abed employs a hybrid strategy that combines the PSO (PSO) algorithm and (NIM) approaches. He accomplishes what he refers to as “optimal parameter estimation” for nonlinear equations (PSO-NIM). His experiments indicate that using a fitness function that is appropriate for the task improves the optimal parameters greatly. This approach is also more accurate and efficient than the old NIM method [6]. Power systems are subject to disruptions due to their nature. Overloading and even unexpected occurrences with higher effect might result from these disruptions. In severe instances, load shedding is used as a last resort to mitigate the effects of an emergency, and its activation is required to prevent system failure. Load shedding systems, on the other hand, rarely perform as intended, resulting in excessive or insufficient load shedding. Cruz et al. presented a load reduction management strategy for medium voltage distribution systems based on PSO to overcome this challenge (PSO). This improvement is intended to reduce the amount of load that must be turned off. Safe operating margins for the loads and voltages of the system components are among the constraints of the optimization issue. He went with heuristic optimization techniques since they are the online foundation for issue resolution [7]. The tongue is employed as an early indicator for illness diagnosis in Greek, Western, and Chinese cultures. Tongues can be used to detect illnesses in a noninvasive approach in the medical field. Diseases and illnesses can cause a wide range of symptoms on the tongue. As a result, Selvarani and Suresh suggested that tongue thermal imaging be used to detect diabetes. A PSO (PSO) algorithm was used to cluster thermally active pixels with similar intensities. For both normal and diabetic patients, the aggregated tongue temperature area showed dramatic changes. The study involved 25 normal people and 25 people with type 1 diabetes. And the accuracy of this method in diagnosing diabetes is 86% [8]. However, the shortcomings of these studies are that the PSO algorithm has low performance, cannot continue to optimize, and the accuracy is not high enough to effectively solve discrete and combinatorial optimization problems.

## 3. Optimization Method of Intelligent Education Based on Particle Swarm Algorithm

As for the introduction of PSO, PSO is a random search algorithm proposed from the research on bird flock foraging [9]. The PSO algorithm is a process of simulating the flock of birds looking for food, and each bird in the flock is regarded as a particle of the population in the algorithm. That is, a possible solution to the problem of minimum peak-valley difference is solved through the motion of particles. These birds are mobile when looking for food. By changing the position and speed of their flight, they keep approaching food until they find it, and the same is true for PSO. The particle keeps approaching the optimal solution by updating its position and velocity until it is found [10].  Figure 1 is a basic block diagram of the PSO algorithm flow.

The PSO algorithm's fundamental frame diagram, which can be broken down into the following steps: (1) initialization: it creates particle speed and position at random. (2) Population evaluation: value of fitness of each population's particles is calculated. (3) Learning sample updates: for each population's particles, it compares its fitness value to value of fitness corresponding to its ideal historical location (pbest). Replace pbest with the current particle location if it is larger than value of fitness of pbest. Value of fitness of pbest is then compared to value of fitness of the population's ideal particle location (gbest). Similarly, if it is a big one, use pbest position instead of gbest. (4) Particle revision: it updates the speed and position of particles in the population.

### 3.1. PSO Algorithm

#### 3.1.1. Introduction to PSO Algorithm

The population of *m* particles in the PSO algorithm “flies” in the *n*-dimensional solution space to find the best solution, and the search is iterative [11]. Position and velocity are two attributes of each population's particles. Each position of the particle in the solution space corresponds to a possible solution to the problem to be optimized. Individual particles have memory function. It can record the optimal position that it has experienced during the search process (called individual optimal position *Q*_*i*_, *i* represents the particle number) and ideal position for all particles(called overall optimal position *Q*_*p*_). The original PSO algorithm has shortcomings and cannot guarantee algorithm convergence. The commonly used PSO algorithm is an improved version with inertial weights [12]. In each iteration of the PSO algorithm with inertia weights, the velocity *V*_*ij*_ and position *X*_*ij*_ of the *j*th dimension of particle *i* are updated according to the following expressions:

(1) $$\begin{array}{c} V_{ij}\left(T+1\right)=\varpi V_{ij}\left(T\right)+G_{1}U_{1j}\left(T\right)\left(Q_{ij}-X_{ij}\left(T\right)\right)+G_{2}U_{2j}\left(T\right)\left(Q_{pj}-X_{ij}\left(T\right)\right), \end{array}$$

(2) $$\begin{array}{c} X_{ij}\left(T+1\right)=X_{ij}\left(T\right)+V_{ij}\left(T+1\right), \end{array}$$

where *T* represents iteration's numbers, *i*=1,2,…, *n*_*g*_, *j*=1,2,…, *n*, *n*_*g*_ is used to represent the population's particle number, N represents the dimension of the solution space, *ω* is the weight of inertia, *G*_1_ and *G*_2_ are coefficients of acceleration, and *U*_1*j*_ and *U*_2*j*_ are random numbers that are distributed uniformly in [0, 1] [13]. Formula (1) consists of 3 parts. Part 1 is the “cricket” part, which means that the particles preserve their earlier velocity. Part cognitive, which is second part, is utilised to represent thinking of the particle itself, so 1 is also called the cognitive coefficient. Part 3 is the “Social” part. It represents the mutual cooperation and information sharing between particles, so 1 is also called the social coefficient.

Steps of the standard algorithm (PSO): (1) let *t* = 0, which initializes the position *x*_*i*_(0) and velocity *v*_*i*_(0) of each population's particles; (2) it calculates value of fitness *f*(*x*_*i*_(*t*)) of each particle; (3) it updates the individual optimal position *Q*_*i*_ of each particle; (4) it updates the overall optimal position *Q*_*p*_; (5) it updates the position of each particle according to formula (1). If the particle velocity is out of bounds, the out-of-bounds processing is performed; (6) it updates the position of each particle according to formula (2). If the particle position is out of bounds, the out-of-bounds processing is performed; and (7) *t* = *t* + 1, if the end condition is met, the algorithm ends; otherwise, go to (2).

#### 3.1.2. Topological Structure Research of PSO Algorithm

Researchers have estimated the performance of the PSO algorithm for graph topology and random neighborhoods in the literature. When the population size is 20 particles, the PSO algorithm with the neighborhood structure of 5 particles performs better. The common population topology of the PSO algorithm is shown in Figure 2. This topology of Figure 2(e) can make the PSO algorithm perform better than the full topology as well as other topologies [14].

#### 3.1.3. Stagnation Detection PSO Algorithm

For the LocalBest PSO algorithm of Ring neighborhood topology, the update expression of the *i*th particle velocity and position in each iteration is as follows:

(3) $$\begin{array}{c} V_{i\;d}\left(T+1\right)=\omega V_{i\;d}\left(T\right)+G_{1}U_{1\;d}\left(T\right)\left(Q_{i\;d}\left(T\right)-X_{i\;d}\left(T\right)\right)+G_{2}V_{i\;d}U_{2\;d}\left(T\right)\left(Q_{i\;d}\left(T\right)-X_{i\;d}\left(T\right)\right),\\ X_{i\;d}\left(T+1\right)=X_{i\;d}\left(T\right)+V_{i\;d}\left(T+1\right). \end{array}$$

The *Q*_*p*_ in the traditional PSO algorithm formula is replaced by the individual neighborhood optimal *Q*_1_. It is expected to weaken the influence of the global optimal particle and enhance the ability of PSO. In the formula, *i*=1,2,…, *m*, *d*=1,2,…, *D*, *D*-dimensional vectors *X*_*i*_(*T*) and *V*_*i*_(*T*) are the position and velocity of particle *i* at time *t*, respectively. *Q*_*i*_ is the individual optimal position that particle *i* has experienced, and *Q*_*p*_ is the global historical optimal position that all neighborhood individuals have experienced. *ω* is the inertia weight, *G*_1_, *G*_2_ is the acceleration coefficient, and *U*_1  *d*_, *U*_2  *d*_ is a random number uniformly distributed in [0, 1] [15].

### 3.2. Radial Basis NN Based on PSO Algorithm

#### 3.2.1. RBF NN Model

RBF is a feed-forward NN with layers preferably three [16]. Input layer consist of one node (which is source), whereas 2^nd^ is submerged layer. Hidden unit's numbers are determined by the situation's requirements. The hidden unit's function of the transformation RBF, which is a function (particularly non-negative and nonlinear) that decays and is radially symmetric to the center point. Output layer is represented by 3^rd^ layer that reacts to the implications of input patterns. The transition from input to hidden layer space is nonlinear. There is a linear transition from the space of the concealed layer to the space of output layer.

The activation function of the RBF NN is based on the radial basis function. It is frequently referred to as a monotonic procedure of the distance measure, i.e., Euclidean, between any point in space and a certain center [17]. Multiple quadratic, thin plate spline, and inverse multiple quadratic functions are examples of radial basis functions.

(*ϕ*(*x*)=(*x*^2^+*c*)^−(1/2)^), and Gaussian function (*ϕ*_*j*_(*x*)=exp(−(‖*x* − *c*_*j*_‖/2*σ*_*j*_^2^))). Figure 3 depicts the RBF NN's neuron topology. The basic idea is to construct the hidden layer space using the RBF function as the hidden unit's “base.” This allows the input vector to be immediately mapped into the latent space (i.e., without the need of weights). The hidden layer space mapping's output space is linear. That is, the output of the network is a linearly weighted sum of the outputs of the hidden units. In most circumstances, the network's weight may be computed easily by solving the linear equation. As a result, learning is significantly expedited, and concerns with local minima are avoided. In most circumstances, the weight of the network may be solved using a simple linear equation. As a result, learning is significantly expedited, and concerns with local minima are avoided.

#### 3.2.2. Learning Technique of RBF NN

The development of the RBF NN type has given NN research and application a new lease on life. The RBF NN is a three-layer feedforward network with a single hidden layer that contains nodes with radial basis functions. The structure of the RBF NN is shown in Figure 4.

According to the RBF NN's network structure, the RBF NN learning method must resolve three different measure: basic function's center, weight and variance from hidden to output layer, respectively. As a result, learning RBF NNs is frequently divided into two steps. In the first step, the basis function's center and variance are established, and in the second phase, the weights from the hidden layer to the output layer are computed. RBF NN learning methods are divided into two categories: central supervised learning algorithms and central unsupervised learning algorithms are two types of central learning algorithms.

*(1) Central Unsupervised Learning Algorithm*. There are many kinds of unsupervised learning algorithms at the center of RBF NN, such as random selection center method and K-means clustering algorithm. The premise of randomly picking a fixed center is that the training data are distributed in a way typical of the problem at hand. And it sets the activation function of the hidden layer unit as a radial basis function whose width is a fixed value. The center position can then be randomly selected from the training data set. For the activation function of the radial base layer, an isotropic Gaussian function can be used. Its standard deviation is determined according to the center walk [18]. Then a radial basis function centered at *S*_*i*_ is defined as

(4) $$\begin{array}{c} L\left({\left\|X-S_{i}\right\|}^{2}\right)=\text{EXP}\left(-\frac{K}{D_{\max}^{2}}{\left\|X-S_{i}\right\|}^{2}\right),\;i=1,2,\ldots ,K, \end{array}$$

where *K* represents the center's number and *D*_max_ represent distance (maximum) between the selected centers. The width of the radial base Gaussian function is fixed to $\sigma =\left(D_{m}/\sqrt{2m}\right)$. This choice of *σ* makes the shape of the Gaussian function moderate, neither too sharp nor too flat. The determination of the weights of the output layer can use the M-P pseudo-inverse learning algorithm. It uses formula *W*=*δ*^+^*D*, where *D* is the chosen retort vector, *δ*^+^ is the inverse of matrix *δ*, and *δ* is determined by

(5) $$\begin{array}{c} \delta =\left\{\chi_{ij}\right\},\\ \chi_{ij}=\text{EXP}{\left(-\frac{m}{D_{m}^{2}}\left\|X_{j}-S_{i}\right\|\right)}^{2},\;\left(j=1,2,\ldots ,m\right). \end{array}$$

The pseudo-inverse of matrix *δ* can be calculated as

(6) $$\begin{array}{c} \delta^{+}={\left(\delta^{t}\delta \right)}^{-1}\delta^{t}. \end{array}$$

*(2) Central Supervised Learning Algorithms.* A supervised learning algorithm is used for the center and output weights of the RBF NN. It can improve the generalization performance of RBF NN [19]. This assumes that the network output is one-dimensional, using the following sum-of-squares cost function:

(7) $$\begin{array}{c} E=\frac{1}{2}\sum_{2}^{C}f_{i}^{2}. \end{array}$$

Here, *C* is the number of training samples and *f*_*i*_ is the error of the network output.

It determines the RBF network's parameters, such as the RBF's center, width, and weights. As a result, the cost function described above is exceedingly minimal. The gradient descent approach to tackle the aforementioned issue has the following optimization formula [20] if the Gaussian function is employed as the radial basis function. The error function's partial derivative with regard to the weights is

(8) $$\begin{array}{c} \frac{\partial G}{\partial V_{j}}=-\sum_{i=1}^{C}f_{i}\phi_{j}. \end{array}$$

Derivative (partial in this case) of the error procedure with the respective center of the RBF is

(9) $$\begin{array}{c} \frac{\partial G}{\partial V_{j}}=-\sum_{i=1}^{C}f_{i}\omega_{j}\frac{\partial \phi_{j}}{\partial V_{j}}. \end{array}$$

Derivative (partial in this case) of the error function with the respective width is

(10) $$\begin{array}{c} \frac{\partial G}{\partial \sigma_{j}}=-\sum_{i=1}^{C}f_{i}\omega_{j}\frac{\partial \phi_{j}}{\partial \sigma_{j}}. \end{array}$$

Derivative (partial in this case) of the RBF function with the respective center is

(11) $$\begin{array}{c} \frac{\partial \phi_{j}}{\partial V_{j}}=2\phi_{j}\left(X_{i}\right)\frac{\left\|X_{i}-V_{j}\right\|}{\sigma_{j}^{2}}. \end{array}$$

Derivative (partial in this case) of the RBF function with the respective width is

(12) $$\begin{array}{c} \frac{\partial \phi_{j}}{\partial \sigma_{j}}=2\phi_{j}\left(X_{i}\right)\frac{\left\|X_{i}-V_{j}\right\|}{\sigma_{j}^{2}}. \end{array}$$

Then, the update formula of the hidden layer center, width and output layer weight of the RBF network is as follows:

(13) $$\begin{array}{c} V_{j}\left(K+1\right)=V_{j}\left(K\right)+\Delta V_{j}=V_{j}\left(K\right)+\varepsilon_{1}\frac{\partial E}{\partial V_{j}},\\ \sigma_{j}\left(K+1\right)=\sigma_{j}\left(K\right)+\Delta \sigma_{j}=\sigma_{j}\left(K\right)+\varepsilon_{2}\frac{\partial E}{\partial \sigma_{j}},\\ \omega_{j}\left(K+1\right)=\omega_{j}\left(K\right)+\Delta \omega_{j}=\omega_{j}\left(K\right)+\varepsilon_{3}\frac{\partial E}{\partial \omega_{j}}. \end{array}$$

Here, *ε*_1_, *ε*_2_, and *ε*_3_ are the learning rate, which can take different values.

### 3.3. RBF NN Based on PSO Algorithm

#### 3.3.1. P-RBF Algorithm Idea

RBF NN has the property of global approximation and is a forward NN with good performance [21]. However, whether the approximation performance of RBF NN can achieve the best effect is closely related to the determination of its structure. When it uses the RBF NN for function approximation, it can easily lead to the “curse of dimensionality” problem [22].

In this paper, the PSO algorithm is used to adjust the training method of this RBF NN, so that the hidden layer's neuron's numbers unit can be arbitrarily set. Adjust to better achieve the training effect. We call this improved algorithm the P-RBF algorithm, which can effectively reduce the hidden layer's neuron's numbers. The algorithm idea is as follows. First, since the function approximation output layer has only one output, its network structure is shown in Figure 5.

Then there are the weights, each of which corresponds to a certain neuron in the hidden layer. Assuming that the input of the network is *X*={*x*_1_, *x*_2_,…, *x*_*n*_}, hidden layer's number units is *m*, and *D*(*i*=1,2,…, *m*) represents the center of the *i*th RBF, the output of the hidden layer unit *Q*(*i*=1,2,…, *m*) is

(14) $$\begin{array}{c} Q_{i}=C_{i}\left(\left\|X-D_{i}\right\|\right). \end{array}$$

It sets the weight between the *i*th neuron in the hidden layer and the output neuron to be *ϖ*_*i*_. Then the output of the output unit is

(15) $$\begin{array}{c} Z=\sum_{i=1}^{m}\varpi_{i}Q_{i}. \end{array}$$

Combining the above formula, the input-output relationship of the network can be obtained as

(16) $$\begin{array}{c} Z=\sum_{i=1}^{m}\varpi_{i}C\left(\left\|X-D_{i}\right\|\right). \end{array}$$

The idea of the P-RBF network algorithm is to first determine a smaller number of hidden layer units, and then use the PSO algorithm to optimize the network weights shown in formula (16). After it reaches a certain iterative algebra, if the network error is still large, hidden layer's number units will be increased. It then uses the PSO algorithm to optimize the network weights, and repeats this process until the network target error is reached [23].

The algorithm's particular method is as follows: (1) it determines the network's hidden layer unit's growth step size l, the radial basis function's width, and the network's goal error. (2) It starts with 0 neurons and works its way up. (3) It uses the Euclidean distance between the target output and the actual output of the network as the PSO algorithm's evaluation function and stops after *n* iterations; it uses the input vector with the largest error in the network as the weight vector to generate a new hidden layer neuron and stops when hidden layer's number neurons increases by l; it uses the Euclidean distance between the target output and the actual output of the network as the evaluation function of the PSO algorithm and stops after *n.* If the network output error does not approach the goal error, it advances to (4), otherwise to (6); (4) it raises hidden layer's number of neurons by utilising the input vector with the biggest mistake as the weight vector to construct a new hidden layer neuron, and it stops when the number of neurons grows. (5) It iterates the PSO method to re-optimize the network weights, checking whether the network output error is less than the goal error; if not, it continues. If not, the algorithm moves on to step (4), otherwise to step (6); (6) The technique ends when the network goal error is reached.

#### 3.3.2. Expal Analysis

It is found through Exps that when approximating the triangular sine function *Y* = sin*x*, if the input vector is in a period of 2*π*, when target neurons in the hidden layer is set to 10, the approximation of the trigonometric function by the network is not very good [24]. The difference between the RBF network's output and the original function curve is still fairly considerable, as seen in Figure 6. When the hidden layer's number of neurons approaches 20, the network output error can be reduced to a very tiny value. As demonstrated in Figure 7, the curve learned by this network may almost exactly match the original sine curve. When the input vector period is increased to 4 and hidden layer's number units is increased to 10, the error becomes quite big, as illustrated in Figure 8. When hidden layer's number units is 20, there is still an inaccuracy, as seen in Figure 9. It can be seen that the P-RBF algorithm can effectively reduce the hidden layer's neuron's numbers and reduce the waste of resources.

## 4. Design and Analysis of the Intelligent Education Personalized System

### 4.1. Functional Structure Design

The functional structure design of the personalized distance education learning management system is based on the use case model and participant model of demand analysis. It divides the system into modules such as system management, information release management, teaching resource management, auxiliary management, and personalized learning management [25]. The specific functional structure is shown in Figure 10.

### 4.2. Comprehensive Performance Analysis of Online Learning Path Planning

In order to verify the performance of learning path planning based on the core algorithm of NBPSO from multiple perspectives, five groups of Exps are implemented in this part. The Expal parameters are shown in Table 1.

The difference in the number of knowledge points will affect the accuracy and matching degree of intelligent education path planning. The number of learners also affects the speed and accuracy of learning path planning. In the first three Exps, different knowledge points were set to compare the Expal effects when the learners were the same. In these three sets of Exps, the corresponding total number of learning resources are 250, 500, and 1000, respectively. In the latter two Exps, different learners were set to compare the Expal results under the same knowledge points.

### 4.3. Expal Results and Analysis

Table 2 is the mean and variance obtained after each core algorithm is run independently for 30 times. The data shown in Table 2 are the mean and variance of the fitness function values constructed in this chapter. It can be seen from the mean data that among the four core algorithms, the mean value and variance of the difference between the two obtained by the NBPSO core algorithm proposed in this chapter are the smallest. This indicates that the planned learning path is more accurate and more in line with the learner's characteristics. It can be seen from the variance data that the variance data obtained by the path planning method with NBPSO as the core algorithm is also the smallest among all the planning methods. This shows that the proposed method has better stability in learning path performance and better service quality.

From the above Expal data, it can be concluded that the basic BPSO core algorithm used in online learning path planning has better convergence performance and can plan a better learning path. But the optimization time of BPSO core algorithm is long. The core algorithm of NBPSO initializes the particle population through logistic map and uses the disturbance term and replacement strategy to enhance the population diversity to improve the convergence accuracy and speed of the algorithm. Its convergence performance is much higher than the other four comparison core algorithms.

## 5. Discussion

In the era of “Internet +” and artificial intelligence, intelligent education and learning will become one of the mainstream learning modes. Intelligent education services will become an important feature of online learning in the future. The increasing size of online learning groups and the demand for personalized services also bring challenges to online learning services. Intelligent education learning has gradually evolved into a learner-centered, emphasizing universal and personalized learning technology. Therefore, the use of intelligent computing technology is to carry out learner learning behavior analysis. It studies group learning behavior patterns and builds an analysis model of learner behavior. It also deeply understands how learners behave in different scenarios. It explores a multidimensional feature model that can fully describe the learning state of learners and studies its utility. This is of great significance to the research on online intelligent learning in the context of the “Internet +” era.

This paper has carried out some research work on the PSO algorithm in swarm intelligence. But these works are only preliminary attempts to apply intelligent computing technology in the field of learning. The impact of key parameters on algorithm search performance and the analysis of algorithm computational complexity remain to be further studied. At the same time, it also considers that the optimization and selection of optimal or suboptimal feature subsets require higher computational cost factors by using the search algorithm based on the objective function. It explores the application mode of cutting-edge artificial intelligence technologies such as machine learning and deep learning in the field of personalized learning. It carries out research on human-machine collaborative adaptive learning methods and learning platforms, interactive learning models based on situational awareness and their environment construction, and research on online learning feedback and evaluation methods and tools based on machine learning. These are all good research directions.

The full mining and innovative application of educational big data can realize the visualization of online learning process, the automation of learning analysis, and the prediction of learning results. It builds an online learning community based on educational big data and promotes the in-depth development of intelligent education applications. This provides an intelligent teaching service environment for the improvement of teaching quality. Smart education driven by big data not only provides us with scientific macro-characteristics and laws but also can customize micro-positioning and precise guidance according to individual characteristics of learners. This effectively solves the problems of deep-level learning behavior analysis and mining and adaptive intelligent interactive learning in complex human-technical interaction environment. Therefore, it is also very meaningful to carry out research and application of key technologies of educational big data for online learning.

## 6. Conclusion

The essence of intelligent education is the process of learners' self-construction of knowledge and continuous improvement of personality under the environment of intelligent learning. It applies artificial intelligence technology to the field of education and provides a series of online learning scenarios and learning activities for learners to complete the process. As for leading the development of intelligent education, it is a research topic worthy of exploration and practice. In this paper, the swarm intelligence PSO algorithm is applied to the field of intelligent education and learning, and exploratory research work is carried out from the perspective of technical performance analysis. The research results mainly focus on the model, method theoretical research and simulation Exp level of technology serving learning. It also needs to continuously improve and optimize the research results through online learning and practical application environment verification. In a word, the information technology represented by the Internet is developing rapidly and changing with each passing day. Facing the major challenges of educational reform, the requirements for scientific education and precise services are constantly increasing. The exploration of smart education driven by data continues to move forward. In a word, the information technology represented by the Internet is developing rapidly and changing with each passing day. Facing the major challenges of educational reform, the requirements for scientific education and precise services are constantly increasing. The exploration of smart education driven by data continues to move forward. Systematic change and cross-industry collaboration are the inevitable way to promote online intelligent learning research and nurture the future education innovation ecosystem. Therefore, it is only necessary to continuously track the cutting-edge technology of artificial intelligence and have the courage to explore and try new models of technical service education. Only by concentrating on new methods of technical service education can we do a better job of smart education research services.

## Figures and Tables

**Figure 1:** PSO flow chart.

**Figure 2:** Common population topology of the PSO algorithm.

**Figure 3:** Radial basis neuron model.

**Figure 4:** RBF NN structure.

**Figure 5:** An output RBF network model.

**Figure 6:** Input range 0–2*π*, and the number of hidden layer units is 10.

**Figure 7:** Input range 0–2*π*, and the number of hidden layer units is 20.

**Figure 8:** Input range 0–4*π*, and the number of hidden layer units is 10.

**Figure 9:** Input range 0–4*π*, and the number of hidden layer units is 20.

**Figure 10:** Functional structure diagram of the personalized education learning management system.

**Table 1:** Learning path planning problem model parameters.

Parameter name	Exp 1	Exp 2	Exp 3	Exp 4	Exp 5
*A*_*M*_	100	150	300	150	150
*B*_*N*_	10	10	10	10	10
*C*_*K*_	1	1	1	10	15
*D*_*K*_	The capability level is divided into five levels, which are initialized randomly				
*E*_*MN*_	Matching degree between the *m*th knowledge point and the *n*th learning resource				
*F*_*nr* ^*i*^ *lr*_*j*__	Learning cost of completing the *i*th to *j*th learning resources				
*J*_*N*_	The difficulty is divided into five levels, which are initialized randomly				

**Table 2:** Expal simulation results.

Core algorithm		Exp 1	Exp 2	Exp 3	Exp 4	Exp 5
BPSO	Avg	2.24*E* + 02	6.58*E* + 02	1.59*E* + 03	5.76*E* + 03	1.35*E* + 04
	Var	2.89*E* + 02	1.07*E* + 03	5.22*E* + 03	5.69*E* + 04	2.08*E* + 05

RPSO	Avg	6.05*E* + 02	1.38*E* + 03	2.86*E* + 03	7.55*E* + 03	1.62*E* + 04
	Var	5.89*E* + 02	3.19*E* + 03	9.06*E* + 03	7.05*E* + 04	3.01*E* + 05

VBPSO	Avg	5.78*E* + 02	1.05*E* + 03	2.81*E* + 03	7.59*E* + 03	1.64*E* + 04
	Var	7.25*E* + 02	1.89*E* + 03	1.06*E* + 04	7.62*E* + 04	2.88*E* + 05

NBPSO	Avg	1.13*E* + 02	1.59*E* + 02	1.89*E* + 02	3.88*E* + 02	6.07*E* + 02
	Var	1.88*E* + 02	3.58*E* + 02	5.01*E* + 02	1.32*E* + 03	1.63*E* + 03

## Data Availability

No data were used to support this study.

## References

[1] Chau K. Y., Law K. M. Y., Tang Y. M. (2021). Impact of self-directed learning and educational technology readiness on synchronous E-learning. *Journal of Organizational and End User Computing*.

[2] Chen H., Fang L., Fan D. L., Huang W., Zeng L. (2019). PSO algorithm with mutation operator for particle filter noise reduction in mechanical fault diagnosis. *International Journal of Pattern Recognition and Artificial Intelligence*.

[3] Durga V. S., Jeyaprakash T. (2021). Predicting academic performance of deaf students using feed forward neural network and an improved PSO algorithm. *Webology*.

[4] Daryina A. N., Prokopiev I. V. (2021). Parametric optimization of unmanned vehicle controller by PSO algorithm. *Procedia Computer Science*.

[5] Mouachi R., Jallal M. A., Gharnati F., Raoufi M. (2020). Multiobjective sizing of an autonomous hybrid Microgrid using a multimodal delayed PSO algorithm: a case study of a fishing village. *Computational Intelligence and Neuroscience*.

[6] Abed K. A. (2020). Solving Kuramoto–Sivashinsky equation by the new iterative method and estimate the optimal parameters by using PSO algorithm. *Indonesian Journal of Electrical Engineering and Computer Science*.

[7] Cruz L. M., Alvarez D. L., Al-Sumaiti A. S., Rivera S. (2020). Load curtailment optimization using the PSO algorithm for enhancing the reliability of distribution networks. *Energies*.

[8] Selvarani A., Suresh G. R. (2020). Preclinical diagnosis of diabetes with tongue infrared thermography and PSO algorithm. *Medico-Legal Update*.

[9] Hannan M. A., Akhtar M., Begum R. A., Basri H., Hussain A., Scavino E. (2018). Capacitated vehicle-routing problem model for scheduled solid waste collection and route optimization using PSO algorithm. *Waste Management*.

[10] Nayak J. R., Shaw B., Sahu B. K. (2017). Load frequency control of hydro-thermal power system using fuzzy PID controller optimized by hybrid DECPSO algorithm. *International Journal of Pure and Applied Mathematics*.

[11] Shukur W. A., Jabbar K. K. (2018). Information hiding using LSB technique based on developed PSO algorithm. *International Journal of Electrical and Computer Engineering*.

[12] Mahmoud A. (2021). Salam, Intelligent system for IoT botnet detection using SVM and PSO optimization. *Journal of Intelligent Systems and Internet of Things*.

[13] Hemavathi P., Nandakumar A. N. (2018). Novel scheme for minimal iterative PSO algorithm for extending network lifetime of wireless sensor network. *International Journal of Electrical and Computer Engineering*.

[14] Kolahi M. R., Nemati A., Yari M. (2018). Performance optimization and improvement of a flash-binary geothermal power plant using zeotropic mixtures with PSO algorithm. *Geothermics*.

[15] Liu C., Wu H., Wang L., Zhang Z. (2017). Tool wear state recognition based on LS-SVM with the PSO algorithm. *Qinghua Daxue Xuebao/Journal of Tsinghua University*.

[16] Khan N. A., Ibrahim Khalaf O., Andrés Tavera Romero C., Sulaiman M., Maharani A. (2022). Application of intelligent paradigm through NNs for numerical solution of multiorder fractional differential equations. *Computational Intelligence and Neuroscience*.

[17] Mahmoodzadeh A., Agahi H., Vaghefi M. (2020). A fall detection system based on the type II fuzzy logic and multi-objective PSO algorithm. *Signal and Data Processing*.

[18] Kavuturu K. K., Narasimham P. (2020). Optimization of transmission system security margin under (N-1) line contingency using improved PSO algorithm. *International Journal on Electrical Engineering and Informatics*.

[19] Tan J., Xu L., Zhang K., Yang C. (2020). A biological immune mechanism-based quantum PSO algorithm and its application in back analysis for seepage parameters. *Mathematical Problems in Engineering*.

[20] Nayak J. R., Shaw B., Sahu B. K. (2020). Hybrid alopex based DECRPSO algorithm optimized Fuzzy-PID controller for AGC. *Journal of Engineering Research*.

[21] Sachdeva K., Aggarwal S. (2021). A hybrid approach for neural network in pattern storage. *Fusion: Practice and Applications*.

[22] Tian S., Li Y., Li J., Liu G. (2020). Robot global path planning using PSO algorithm based on the interaction mechanism between leaders and individuals. *Journal of Intelligent and Fuzzy Systems*.

[23] Shin J. J., Bang H. (2020). UAV path planning under dynamic threats using an improved PSO algorithm. *International Journal of Aerospace Engineering*.

[24] Singh S., Chauhan P., Singh N. J. (2020). Capacity optimization of grid connected solar/fuel cell energy system using hybrid ABC-PSO algorithm. *International Journal of Hydrogen Energy*.

[25] Regis N., Muriithi C. M., Ngoo L. (2019). Optimal battery sizing of a grid-connected residential photovoltaic system for cost minimization using PSO algorithm. *Engineering, Technology & Applied Science Research*.

